The article "lncRNA BZRAP1‐AS1 alleviates rheumatoid arthritis by regulating miR‐1286/COL5A2 axis" was retracted in 2025. Reasons: original data or images not available; unreliable results or conclusions; concerns about the results or conclusions; concerns about the article.

# lncRNA BZRAP1‐AS1 alleviates rheumatoid arthritis by regulating miR‐1286/COL5A2 axis

**DOI:** 10.1002/iid3.558

**Published:** 2021-11-11

**Authors:** Junsong Zhu, Shaoheng Tu, Qunwei Qu

**Affiliations:** ^1^ Department of Pain Medicine Wuhan University of Science and Technology Affiliated Puren Hospital Wuhan Hubei China; ^2^ Department of Traditional Chinese Medicine Wuhan Pulmonary Hospital Wuhan Hubei China

**Keywords:** apoptosis, inflammation, lncRNA, miRNA, proliferation, rheumatoid arthritis

## Abstract

**Background:**

Dysregulation of BZRAP1‐AS1 was associated with immune statuses of cancer or Alzheimer's disease patients, yet little is known about its role in rheumatoid arthritis.

**Methods:**

RT‐qPCR and western blot were applied to assess the expression of indicated expression. CCK‐8 and BrdU proliferation assays were used to measure the proliferation of RA‐HFLS. Apoptosis in RA‐HFLS was evidenced by the alteration of caspase‐3 activity and apoptosis‐related factors. ELISA was performed to detect IL‐6, IL‐1β, and TNF‐α level. Luciferase reporter, RIP, and pull‐down assays were used to confirm the BZRAP1‐AS1/miR‐1286/COL5A2 cascade predicted by bioinformatics analysis.

**Results:**

BZRAP1‐AS1 and COL5A2 were downregulated in RA tissues and RA‐HFLS while miR‐1286 was amplified. Overexpression of BZRAP1‐AS1 reduced the RA‐HFLS proliferation, IL‐6, IL‐1β, and TNF‐α level and induced cell apoptosis while BZRAP1‐AS1 silence produced an opposite effect. Overexpression of BZRAP1‐AS1 reduced the miR‐1286 expression which in turn increased the COL5A2 expression, thereby relieving the excessive proliferation and limited apoptosis in RA‐HFLS.

**Conclusion:**

Our findings suggested that BZRAP1‐AS1 sequestered miR‐1286 and reshaped the COL5A2 expression, thereby suppressed RA‐HFLS proliferation and inflammation, and triggered cell apoptosis, resulting in the attenuation of RA progression.

## 1 INTRODUCTION

Rheumatoid arthritis (RA) is a chronic autoimmune disease characterized by synovitis of the joints.^1^ Prolonged or recurrent episodes of chronic synovitis led to the destruction of cartilage and bone in the joints, resulting in joint deformities and dysfunction, even disability.^2^ The global incidence rate is about 1%. Apart from virus infection and hormonal dysregulation, gene alteration is a predisposing factor of RA.^3^ Therefore, deeper entangling the genetics implicated in RA helps in understanding RA genesis and progression.

Long noncoding RNA (lncRNA) is a subfamily of noncoding RNA containing more than 200nt. It acts as a DNA/RNA/protein‐binding molecule and plays a multifaceted role in biological and physiological processes, including chromatin remodeling, RNA splicing, RNA transcription, and protein transportation.^4^, ^5^ Recent evidence has shown that their dysregulation or mutates are tightly associated with cancer genesis, Alzheimer's disease, and coronary artery disease.^6^, ^7^, ^8^ lncRNAs alterations also can modulate the expression of inflammatory factors and thereby recruit inflammatory and immune cells, underscoring the involvement of lncRNA in autoimmune disorders, including RA.^9^, ^10^ For example, an elevation of lncRNA PICSAR is detected in synovial fluid of rheumatoid arthritis patients.^11^ In vitro and vitro assays demonstrated that upregulated MEG3 can attenuate the inflammatory response in lipopolysaccharide (LPS)‐treated chondrocyte.^12^ In addition, a significantly negative correlation between plasma levels of lncRNA DILC and IL‐6 was shown in RA patients.^13^ As for BZRAP1‐AS1, Wang et al.^14^ found that its knockout in hepatocellular carcinoma cells reduced the proliferation, migration, and angiogenesis of human umbilical vein endothelial cells, thereby retarding cancer progression. BZRAP1‐AS1 correlates with cervical cancer‐immune cell infiltration.^15^ In addition, BZRAP1‐AS1 is a risk locus of Alzheimer's disease and is related with immune‐related traits of this disease.^16^ However, the role in RA remains unraveled.

The gene of Collagen type V alpha 2 chain (COL5A2) is located on chromosome 2q32.2, consisting of 55 exons. This gene is translated into a 145 KDa alpha chain for one of the low abundance fibrillar collagens. In addition to its roles in cancers, Col5a2 has been found to be mutated in Classic Ehlers–Danlos syndrome and ischemic heart disease.^17^, ^18^, ^19^, ^20^, ^21^ More interesting, Gu et al.^22^ applied weighted gene co‐expression network analysis and identified COL5A2 as a hub gene implicated in the pathological process of osteoarthritis.^22^ However, the role of RA has not been previously reported.

In our current work, we examined the differential expressed genes from RA GEO DataSets and established a BZRAP1‐AS1/miR‐1286/COL5A2 axis. Subsequently, the proliferation and apoptosis of RA‐infected human fibroblast‐like synoviocytes cells (HFLS) were evaluated to validate this predicted cascade. Our findings could enrich our understanding of RA progression.

## 2 METHODS

### 2.1 Human tissue samples

Synovial tissues were collected from RA patients and non‐RA individuals undergoing fracture surgery and stored at −80℃ for quantification of indicated genes. Each patient signed informed consent. Ethical approval was granted by the medical ethics committee of Wuhan University of Science and Technology affiliated Puren Hospital.

### 2.2 Cell incubation and transfection

HFLS and RA‐infected HFLS (RA‐HFLS) were obtained from Cell Applications, Inc. All cells were incubated in Dulbecco's modified Eagle's medium containing 10% fetal bovine serum and 1% penicillin/streptomycin in a 5% CO_2_ atmosphere at 37°C. The pcDNA‐BZRAP1‐AS1 vectors, pcDNA‐COL5A2 vectors, BZRAP1‐AS1 siRNA (si‐BZRAP1‐AS1), miR‐1286 mimic/inhibitor, and their corresponding negative controls were delivered into RA‐HFLS using Lipo 3000 transfection reagent (Thermo Fisher Scientific). For BZRAP1‐AS1 or COL5A2 overexpression, the transfected cells underwent a continuous puromycin selection for 7 days and the survival cell clones were kept for next assays.

### 2.3 Reverse transcription‐polymerase chain reaction (RT‐qPCR)

RNA purification from RA tissues, RA‐HFLS, or HFLS was implemented using TRIzol reagent (Sigma‐Aldrich). MiR‐Quant TaqMan microRNA cDNA Synthesis Kit (Beijing Baiaolaibo Technology Co., Ltd.) and BeyoRT III First‐Strand Synthesis Kit (Beyotime) were applied for synthesis of cDNA from 2 μg total RNA. The real‐time PCR was performed on One Step RT‐qPCR KitABI 7900 HT Fast (Applied Biosystems) with One Step RT‐qPCR Kit (Sangon Biotech). Data were normalized to GAPDH and analyzed by 2^−∆∆Ct^ method. The primers are listed in Table 1.

**Table 1:** PCR primers used in this study

Gene	Primer type	Sequence
BZRAP1‐AS1	Forward	5′‐CTGAATCTCGCTTGATCGT‐3′
	Reverse	5′‐GAGTAGTCGGAAAGGATGC‐3′
TPTEP1	Forward	5′‐AGCCGCAGACAAAAGACCTCGG‐3′
	Reverse	5′‐CCACCAAACAGGCTTCGTGTGA‐3′
LEF1‐AS1	Forward	5′‐AAGGACGAGAGAAAAGCAC‐3′
	Reverse	5′‐CACACAAAGGGGAAGACC‐3′
COL5A2	Forward	5′‐CAGAAGCCCAG ACGTATCG‐3′
	Reverse	5′‐GGTGGTCAGGCACTTCAGAT‐3′
U6	Forward	5'‐TTATGGGTCCTAGCCTGAC‐3‐3′
	Reverse	5'‐CACTATTGCGGGTCTGC‐3'−3′
GAPDH	Forward	5′‐CCTGGCCAAGGTCATCCATG‐3′
	Reverse	5′‐GGAAGGCCATGCCAGTGAGC‐3′

### 2.4 Western blot

Cells were treated by RIPA lysis buffer (Applygen) and centrifuged. Lysate supernatants were harvested and quantified using a BCA kit (Beyotime). 10 µg of protein was separated by 10% sodium dodecyl sulfate–polyacrylamide gel electrophoresis and electrophoresed to polyvinylidene fluoride membrane which was subsequently blocked with 10 ml blocking solution for 1 h. Anti‐Bcl‐2 antibodies, anti‐Bax antibodies, anti‐pro‐caspase‐3 antibodies, anti‐Cleaved caspase‐3 antibodies, and anti‐actin antibodies were added and incubated with membrane overnight at 4°C following another 1 h incubation with the indicated secondary antibodies at room temperature. Blots were visualized by ECL solution and developed in an X‐ray film.

### 2.5 Cell proliferation assay

Cell proliferation was assessed by Cell Counting Kit‐8 (CCK‐8) assays and BrdU assays. For CCK‐8 assay, For CCK‐8 detection, cells were maintained in a 96‐well plate for 24 h. The 20 μl CCK‐8 solution was coincubated with cells for additional 0, 24, 48, and 72 h. The plates were measured at 450 nm. For 5'‐Bromo‐2‐deoxyuridine (BrdU) detection, the logarithmic‐phase cells were treated with 10 μl BrdU for 30 min before being fixed by 4% formaldehyde fixative and blocked with 3% bovine serum albumin. Following, the BrdU‐incorporated cells were detected using a BrdU In‐Situ Detection Kit (BD Biosciences) according to the manual.

### 2.6 Assessment of caspase −3 activity

Detection of caspase‐3 activity was done with a caspase‐3 Activity Assay Kit (Beyotime) as instructed in the kit manual. In brief, 10 μl cell lysates were treated by Apo‐ONE caspase‐3 reagent. After 2 h cell incubation, absorbance was read at 405 nm.

### 2.7 Enzyme‐linked immunosorbent assay (ELISA)

After transfection, RA‐HFLS culture supernatant was collected and diluted for subsequent experiments. Relative cytokine concentrations of TNF‐α, IL‐6, and IL‐1β were evaluated using commercial ELISA kits (R&D Systems). The absolute concentrations of the cytokines shown in each dish were calculated by the standard curve method.

### 2.8 Luciferase reporter assay

The wild‐type luciferase reporter constructs (BZRAP1‐AS1‐WT and COL5A2‐WT) and corresponding mutant vectors (BZRAP1‐AS1‐MUT and COL5A2‐MUT) were generated through fusing the sequence of miR‐1286 target site or mutation into luciferase reporter vector pGL3. The resulted luciferase plasmids were transfected into RA‐HFLS along with miR‐1286 mimic or NC for 48 h. The luciferase activity was evaluated through the Promega Luciferase Assay System.

### 2.9 RNA immunoprecipitation (RIP)

A RNA Immunoprecipitation Kit (Millipore Sigma) was applied to determine the association of BZRAP1‐AS1 and miR‐1286 with protein A/G magnetic beads. The RA‐HFLS were lysed by sonication, and the supernatant was amassed through centrifugation and underwent. Meanwhile, the magnetic beads were resuspended in RIP wash buffer and incubated with anti AGO2 or anti IgG antibodies for 30 min. The resulted magnetic bead‐antibody complex was added into the prepared supernatant sample at 4°C. The next day, the precipitate was collected and treated with Proteinase K at 55°C for 30 min. The supernatant was collected for RT‐qPCR analysis.

### 2.10 RNA pull‐down

Biotin‐labeled miRNA (Bio‐miR‐388‐3p, Bio‐miR‐127‐5p, Bio‐miR‐1286, bio‐miR‐1301‐3p, or Bio‐ NC) (Xi'an, Qiyue Biotech, Co. Ltd.) were introduced into RA‐HFLS. At 48 h posttransfection, the cell lysates were collected for incubation with the magnetic beads as above‐mentioned and prepared for RNA isolation and quantification of COL5A2 mRNA.

### 2.11 Statistical analysis

GraphPad Prism version 8 was employed to analyze the results showed as mean ± *SD*. Unpaired *t* test was adopted to analyze the measurement data from two groups, analysis of variance for comparisons of data among multiply groups. *p* < .05 was considered significant

## 3 RESULTS

### 3.1 lncRNA BZRAP1‐AS1/miR‐1286/COL5A2 axis may be related to RA

GSE94519 from GEO DataSets is the lncRNA expression profile involving RA samples and normal samples. With *p* < .05 and log_2_FC < −1, the downregulated lncRNAs were screened out. As shown in Figure 1A, the top five downregulated lncRNAs were listed. After detecting the expression levels of the top five lncRNAs in our collected synovial tissues, lncRNA BZRAP1‐AS1 with the lowest expression in RA samples was observed (Figure 1B–F). Therefore, BZRAP1‐AS1 was identified as the lncRNA of our interest. Next, GSE2053 and GSE1919 also from GEO DataSets were mRNA expression profiles involving RA samples and normal samples to select the downregulated genes with *p* < .05 and log_2_FC < −1. It was found that COL5A2 was the only common downregulated gene in GSE2053 and GSE1919 (Figure 1G). To identify the miRNA, miRDB and starBase were used to predict miRNAs binding to BZRAP1‐AS1 and COL5A2, respectively. Finally, four miRNAs (miR‐488‐3p, miR‐1286, miR‐1277‐5p, and miR‐1301‐3p) were overlapped (Figure 1H). The RIP assay and RNA pull‐down assay confirmed that miR‐1286 was the key miRNA that could bind to BZRAP1‐AS1 and COL5A2 (Figure 1I,J). These data suggested that lncRNA BZRAP1‐AS1/miR‐1286/COL5A2 axis may be related to RA.

**Figure 1:** The identification of LncRNA BZRAP1‐AS1/miR‐1286/COL5A2 axis in RA. (A) Top five downregulated lncRNAs in an lncRNA expression profile GSE94519. Selection criteria: *p* < .05 and log_2_FC < −1. (B–F) The expression levels of top five downregulated lncRNAs in RA and normal samples. *p < .05, **p < .001. (G) COL5A2 was the only common downregulated gene in GSE2053 and GSE1919. Selection criteria: *p* < .05 and log_2_FC < −1. (H) Four miRNAs might bind to BZRAP1‐AS1 (predicted by miRDB software) and COL5A2 (predicted by starBase). (I) The miRNA binding to BZRAP1‐AS1 was confirmed by RIP assay. versus anti‐lgG, **p < .001. (J) The miRNA binding to COL5A2 was confirmed by RNA pull‐down assay, versus Bio‐NC, **p < .001

### 3.2 Impact of BZRAP1‐AS1 on RA‐HFLS cell proliferation and apoptosis

Afterward, we further tested the expression level of BZRAP1‐AS1 in RA‐HFLS. BZRAP1‐AS1 was highly expressed in RA‐HFLS in comparison with that in normal HFLS cells (Figure 2A). Next, we controlled the BZRAP1‐AS1 expression by introducing si‐ BZRAP1‐AS1 or pcDNA‐BZRAP1‐AS1 vectors or their NC cells into RA‐HFLS. The outcome from RT‐qPCR showed the successful establishment of the BZRAP1‐AS1 knockdown or overexpressing RA‐HFLS (Figure 2B). Next, the proliferation and apoptosis of RA‐HFLS upon ZRAP1‐AS1 silence or ectopical expression were assessed. As shown in Figure 2C, the BZRAP1‐AS1 knockdown led to higher RA‐HFLS cell proliferation while BZRAP1‐AS1 overexpression caused lower cell proliferation compared with the control group cells. Meanwhile, the rate of BrdU‐incorporating live cells was obviously lessened in the BZRAP1‐AS1‐overexpressing RA‐HFLS while elevated in BZRAP1‐AS1‐silencing RA‐HFLS (Figure 2D). Undoubtedly, the caspase‐3 activity was reduced in the BZRAP1‐AS1 knockdown RA‐HFLS along with increased bcl‐2 and reduced Bax and cleaved‐caspase‐3 expression. The BZRAP1‐AS1 overexpressing RA‐HFLS demonstrated opposite outcome (Figure 2E,F). In addition, ELISA results showed that BZRAP1‐AS1 upregulation inhibited the levels of proinflammatory cytokines IL‐6, IL‐1β, and TNF‐α, while BZRAP1‐AS silence increased the inflammatory levels of RA‐HFLS (Figure 2G). Our data suggested that BZRAP1‐AS1 impaired proliferation and triggered apoptosis in RA‐HFLS.

**Figure 2:** BZRAP1‐AS1 suppresses RA‐HFLS cell proliferation. (A) The relative expression of BZRAP1‐AS1 was measured in the normal and RA affected human FLS cells (RA‐HFLS groups and normal FLS group), versus Normal FLS, **p < .001. (B) The relative expression of BZRAP1‐AS1 in RA‐HFLS I with si‐BZRAP1‐AS1 or pcDNA‐BZRAP1‐AS1 vectors. (C) After transfection for 48 h, the cell proliferation was measured by CCK8 assay at continuous culture for 24, 48, and 72 h. (D) BrdU‐incorporating live cells were detected by EDU proliferation assay. (E) Caspase‐3 activity was examined with a caspase‐3 activity detection kit. (F) The Bcl‐2, Bax, pro‐caspase‐3, and cleaved‐caspase‐3 expression were detected by western blot. (G) The IL‐6, IL‐1β, and TNF‐α level were detected by ELISA. Versus empty vectors, **p < .001; versus Si‐NC, ^#^ *p* < .05, ^##^ *p* < .001

### 3.3 BZRAP1‐AS1 targets miR‐1286 as a miRNA sponge to antagonize miR‐1286

The above‐mentioned results revealed the interplay between BZRAP1‐AS1 and miR‐1286, Therefore the starBase V2.0 was used to explore their interaction pairs. As shown in Figure 3A, the BZRAP1‐AS1 contained 8 complementary bases to miR‐1286. Next, the miR‐1286 mimic and NC were delivered into the RA‐HFLS along with luciferase reporter constructs carrying BZRAP1‐AS1‐wide‐type (WT) and BZRAP1‐AS1‐mutant (MUT). The miR‐1286 mimic transfection induced an increased WT‐mediated luciferase activity while changes were observed in other treatments, suggesting that BZRAP1‐AS1 competitively binds to miR‐1286 (Figure 3B). Considering the mechanism of lncRNA‐miRNA interaction, we further assessed the miR‐1286 expression. As anticipated, the miR‐1286 expression was considerably increased and RA patients and RA‐FLS cells. (Figure 3C,D). More importantly, the BZRAP1‐AS1 overexpression significantly reduced the miR‐1286 expression which can be restored by miR‐1286 mimic (Figure 3E). In addition, the transfection efficiency of miR‐1286 mimic and inhibitor has been identified (Figure 3E). These data indicated that BZRAP1‐AS1 functions as a ceRNA to suppress the expression of miR‐1286.

**Figure 3:** BZRAP1‐AS1 targets miR‐1286 with ceRNA activity. (A) miR‐1286 contained the complementary bases with BZRAP1‐AS1. (B) The luciferase activity on behalf of the molecular binding of BZRAP1‐AS1 and miR‐1286 was examined, versus WT + NC. (C) miR‐1286 level in the RA patients was tested using RT‐qPCR. **p < .001. (D) miR‐1286 level in the RA‐HFLS. Versus Normal HFLS, **p < .001. (E) miR‐1286 level was decreased in the RA‐HFLS transfected or cotransfected with BZRAP1‐AS1 or NC and miR‐1286 mimic/inhibitor and NC. Versus Empty vector, **p < .001, versus Mimic‐NC; ^##^ *p* < .001; versus Mimic+lnc‐OE, ^$$^ *p* < .001

### 3.4 The BZRAP1‐AS1‐mediated inhibition of RA‐HFLS cell proliferation through sequestration of miR‐1286

The next cell proliferation was assessed to determine whether BZRAP1‐AS1 functions in RA‐HFLS through complementarily binding to miR‐1286. Figure 4A demonstrates that miR‐1286 mimic increased cell viability and inhibitor decreased it, BZRAP1‐AS1‐overexpression caused weakened proliferation was reversible in RA‐HFLS accompanied with miR‐1286 mimic. Similarly, the percentage of BrdU positive RA‐HFLS containing miR‐1286 mimic or inhibitor are higher or lower than that of control cells, and the lower proliferation of BZRAP1‐AS1‐overexpressing RA‐HFLS was rescued to the levels comparable to the NC groups by the accompanied transfection of miR‐1286 mimic (Figure 4B). Next, we further assessed the apoptosis‐related factors in RA‐HFLS upon cotransfection with pcDNA‐BZRAP1‐AS1 vectors and miR‐1286 mimic. As shown in Figure 4C, miR‐1286 mimic or inhibitor transfection can weaken or facilitate the caspase‐3 activity. More importantly, it can abrogate the stimulated caspase‐3 activity resulted from BZRAP1‐AS1 overexpression. The effect of BZRAP1‐AS1‐miR‐1286 interplay on RA‐HFLS cell apoptosis was further evidenced by western blots. In addition, transient transfection with exogenous miRNA‐1286 mimic can reduce the Bax and cleaved‐caspase‐3 protein expression in addition to increased expression of Bcl‐2, while inhibitor transfection showed an opposite trend. Likewise, the exogenously overexpressed miRNA‐1286 can offset the capacity of BZRAP1‐AS1 to diminish the Bcl‐2 expression as well as promote the cleaved‐caspase‐3 and Bax protein expression (Figure 4D). Furthermore, ELISA was performed to detect the changes in the regulation of BZRAP1‐AS1‐miR‐1286 on pro‐inflammatory factors. The results showed that the low expression of miR‐1286 inhibited the levels of IL‐6, IL‐1β and TNF‐α, while the overexpression of miR‐1286 increased the levels of pro‐inflammatory factors and reversed the inflammatory effect caused by the upregulated BZRAP1‐AS1 (Figure 4E). Taken together, our findings indicated that the ant‐proliferative capacity of BZRAP1‐AS1 was reversed by miRNA‐1286 action.

**Figure 4:** miRNA‐1286 overexpression antagonizes the anti‐proliferation caused by BZRAP1‐AS1 overexpression. RA‐HFLS were cotransfected with miRNA‐1286 mimic and BZRAP1‐AS1 overexpression vectors. Cell proliferation was assessed by CCK8 (A), BrdU incorporation assays (B). (C) Caspase‐3 activity was measured by caspase‐3 activity assay (*n*  =  3). (D) Western blot analysis of apoptosis‐related proteins. (E) ELISA of IL‐6, IL‐1β, and TNF‐α level. Versus Empty vectors, **p < .001; versus Mimic‐NC, ^#^ *p* < .05; ^##^ *p* < .001; versus mimic + lnc‐OE, ^$^ *p* < .05, ^$$^ *p* < .001

### 3.5 COL5A2 is the target of miR‐1286

MiRNA/target mRNA recognition is necessary for miRNA action. Therefore, we identified the target genes of miR‐1286 by TargetScan and constructed the miR‐1286‐COL5A2 synergistic network (Figure 5A). The miR‐1286‐COL5A2 interplay was further evidenced by the reduced COL5A2‐3'UTR WT luciferase activity in RA‐HFLS resulted by miR‐1286 mimic transfection (Figure 5B). More interesting, we found the diminished expression of COL5A2 was testified in RA tissues and RA‐HFLS (Figure 5C,D). In addition, COL5A2 protein expression was prominently reduced in RA‐HFLS after the miR‐1286 mimic intervention (Figure 5E). Collectively, the downregulated COL5A2 expression is associated with miR‐1286 functionality in RA‐HFLS.

**Figure 5:** COL5A2 is the traget of miR‐1286. (A) The WT‐3′UTR of COL5A2 mRNA was predicted as the target of miR‐1286. versus WT + NC, **p < .001. (B) The mRNA of COL5A2 was identified as the target of miR‐8055 using the luciferase reporter assays. RT‐qPCR was performed to assess the COL5A2 expression in RA tissues (C) and RA‐HFLS (D). **p < .001. (E) Western blot analysis assays using COL5A2 antibodies was carried out to determine the COL5A2 protein in RA‐HFLS transfected with miR‐1286 mimic or inhibitor. versus Mimic‐NC, **p < .001; versus Inhibitor‐NC, ^##^ *p* < .001

### 3.6 COL5A2 overexpression antagonizes the pro‐proliferative activity of miR‐1286 in RA‐HFLS

Subsequently, we explored whether the role of miR‐1286 in RA‐HFLS is COL5A2‐dependent. Figure 6A,B demonstrates that COL5A2 ectopical expression caused a proliferative inhibition of RA‐HFLS, and also abolished the miR‐1286‐stimulated cell proliferation. Furthermore, the introduction of miR‐1286 mimic into COL5A2 ectopically expressed RA‐HFLS nullified the increased caspase‐3 activity caused by COL5A2 overexpression (Figure 6C). Consistently, RA‐HFLS transfected with pcDNA‐COL5A2 vectors can weaken the Bcl‐2 expression and increase Bax, cleaved‐caspase‐3 expression, this alteration in the expressions of apoptosis‐related factors was reversed by the addition of miR‐1286 mimic in RA‐HFLS (Figure 6D). In addition, ELISA revealed that upregulated COL5A2 inhibited the IL‐6, IL‐1β, and TNF‐α level, and this inflammatory inhibitory effect was eliminated by miR‐1286 mimic (Figure 6E). Collectively, miR‐1286 enhanced proliferation and blocked apoptosis through downregulation of COL5A2 expression.

**Figure 6:** miR‐1286 enhanced proliferation and blocked apoptosis through downregulation of COL5A2 expression. RA‐HFLS were transfected with miR‐1286 mimic, mimic NC, pcDNA‐COL5A2 vectors for COL5A2‐overexpression, and pcDNA empty vector or cotransfection with pcDNA‐COL5A2 vectors and miR‐1286 mimic for 48 h. (A) CCK8 assays were employed to assess cell proliferation. (B) BrdU incorporation assays. (C) Caspase‐3 activity was measured by caspase‐3 activity assay (*n*  =  3). (D) Western blot analysis of apoptosis‐related proteins. (E) ELISA of IL‐6, IL‐1β, and TNF‐α level. Versus Empty vectors, *p < .05, **p < .001; versus Si‐NC, ^#^ *p* < .05, ^##^ *p* < .001; versus Mimic + lnc‐OE, ^$^ *p* < .05, ^$$^ *p* < .001

## 4 DISCUSSION

Excessive proliferation of HFLS cells in RA patients is the main reason for joint dysfunction.^23^ Hyperplastic HFLS cells not only excrete various proinflammatory cytokines, chemokines, and growth factors but also possesses transforming properties, which contributes to bone and cartilage erosion and aggravates disease manifestations.^24^ Currently, lncRNAs reportedly modulate HFLS cells survival and cell growth, and the inflammatory response during RA progression.^25^ Herein, BZRAP1‐AS1 competitively binds to an effective miR‐1286 sponge and increases the expression of the miR‐1286 target, COL5A2, thereby impedes RA progression.

Initially, BZRAP1‐AS1 showed lower expression in RA synovial tissues and RA‐HFLS, in comparison with the normal synovial samples and normal HFLS cells, respectively, highlighting its potential implication in RA progression. BZRAP1‐AS1 is an oncogenic lncRNA that drives angiogenesis of hepatocellular carcinoma, meanwhile facilitates tumor cell proliferation, migration, and invasion. However, the effect of BZRAP1‐AS1 on RA‐HFLS has not been clarified.^14^ The outcome of our data found that BZRAP1‐AS1 reduced cell proliferation and triggered cell apoptosis in RA‐HFLS. BZRAP1‐AS1 might be related with immune‐related traits of Alzheimer's disease because its association with mean platelet (thrombocyte) volume.^16^ Furthermore, the high‐BZRAP1‐AS1 cervical cancer patients showed different immune statuses in GSEA.^15^ The immune‐related properties of BZRAP1‐AS1 might further support its role in RA.

There is increasing studies about lncRNAs in competitive regulatory interactions which can titrate miRNA and reshape gene expression. In our present work, miR‐1286 was upregulated in RA tissues and RA‐HFLS. Meanwhile, exogenous expression of miR‐1286 mimic induced proliferation, inflammation, and impedes apoptosis of RA‐HFLS. Previously, the oncogenic and tumor‐suppressive roles of miR‐1286 have been reported. For example, in osteosarcoma, anti‐miR‐1286 inhibitors increase the tumor cell malignant behaviors including proliferation.^26^ On the contrary, miR‐1286 can reverse the inhibited cell migration and invasion caused in lung adenocarcinoma by lncRNA ITINCR.^27^ Therefore, the miR‐1286 might have distinct roles in different tissues. More importantly, our results revealed that BZRAP1‐AS1 directly bound miR‐1286. The miR‐1286 expression in RA tissues or RA‐HFLS showed an opposite trend to BZRAP1‐AS1. Its ectopic expression can relieve the antiproliferative and anti‐inflammatory function of BZRAP1‐AS1. All these results confirm that BZRAP1‐AS1 drives RA‐HFLS cell proliferation by sponging miR‐1286.

MiRNAs exert functions by base pairing to target mRNAs. COL5A2 is a target gene of miR‐1286. Contrary to the downregulated miR‐1286, COL5A2 was upregulated in RA tissues and RA‐HFLS. Undoubtedly, the miR‐1286 mimic transfection weakened the expression of COL5A2 while the miR‐1286 inhibitor transfection boosted COL5A2 expression in RA‐HFLS. In parallel, the COL5A2 overexpression resulted in less proliferative and inflammatory potential, and higher apoptosis levels in RA‐HFLS. Highly expressed COL5A2 can abrogate the boosted proliferation and inflammation, and impede apoptosis caused by miR‐1286 mimic. Therefore, miR‐1286/COL5A2 cascade might be the downstream effectors of BZRAP1‐AS1 in RA progression.

Our investigation has limitations. The sample size was few for the detection of BZRAP1‐AS1, miR‐1286, and COL5A2 expression. Additionally, in vivo experiments are required to affirm the function of BZRAP1‐AS1 in RA.

## 5 CONCLUSION

Conclusively, our findings revealed that BZRAP1‐AS1 impedes the miR‐1286 activity by ceRNA activity and upregulated COL5A2 expression, attenuating RA progression. BZRAP1‐AS1 negatively governed the RA‐HFLS cell proliferation and inflammation, and induced apoptosis. in RA‐HFLS. Thusly, the BZRAP1‐AS1 might function as a promising target for RA diagnosis and intervention.

## CONFLICT OF INTERESTS

The authors declare that there are no conflict of interests.

## AUTHOR CONTRIBUTIONS

Junsong Zhu and Shaoheng Tu conducted the study and collected and analyzed the data. Junsong Zhu designed the study and methods and collected the funds. Shaoheng Tu analyzed and interpreted the data. Qunwei Qu collected materials and resources, conducted literature analysis, and prepared manuscript. Qunwei Qu conducted a literature analysis and prepared the manuscript. All authors read and approved the final manuscript.

## ETHICS STATEMENT

The present study was approved by the Ethics Committee of Wuhan University of Science and Technology Affiliated Puren Hospital (Wuhan, China). The processing of clinical tissue samples is in strict compliance with the ethical standards of the Declaration of Helsinki. All patients signed written informed consent.

## Data Availability

The datasets used and analyzed during the current study are available from the corresponding author on reasonable request.
